RETRACTED

# Association between Perceived Salt Intake and Arterial Stiffness

**DOI:** 10.1155/2022/9072082

**Published:** 2022-07-06

**Authors:** Mengdi Jin, Congliang Miao, Lina An, Li Guo, Xinying Yang, Mengyi Zheng, Jiang Hong, Shouling Wu, Qi Su

**Affiliations:** ^1^Department of Emergency and Critical Care, Shanghai General Hospital, Shanghai Jiao Tong University School of Medicine, Shanghai 200080, China; ^2^Department of Geriatrics, Shanghai General Hospital, Shanghai Jiao Tong University School of Medicine, Shanghai 200080, China; ^3^Department of Cardiology, Shanghai General Hospital of Nanjing Medical University, Shanghai 200080, China; ^4^Department of Cardiology, Shanghai General Hospital, Shanghai Jiao Tong University, Shanghai 200080, China; ^5^Cardiovascular Center, Beijing Tongren Hospital, Capital Medical University, Beijing 100730, China; ^6^Department of Emergency and Critical Care, Shanghai General Hospital, Shanghai Jiao Tong University, Shanghai 201600, China; ^7^Department of Cardiology, Kailuan Hospital, North China University of Science and Technology, Tangshan 063000, China

## Abstract

To explore the association of perceived salt intake (SI) level with arterial stiffness in the community population in northern China. We enrolled participants who completed the health questionnaire, physical examination, and brachial-ankle pulse wave velocity (baPWV) test during 2010-2019 and divided them into <6 g (low SI), 6-10 g (medium SI), and >10 g (high SI) groups based on their daily SI. The influence of SI on baPWV was analyzed using the multivariate logistic regression model. A total of 36324 subjects, aged (49.10 ± 12.57) years with a male to female ratio of 25934 : 10390, met the inclusion criteria and were enrolled. The average baPWV was (1527.73 ± 355.61) cm/s. Logistic regression analysis showed that after adjusting for other confounders, daily SI>10 g (high SI) was a risk factor for arterial stiffness (baPWV ≥1400 cm/s), with the odds ratio (95% confidence interval [CI]) of 1.17 (1.04-1.31). High SI is independently associated with arterial stiffness.

## 1. Introduction

Globally, high salt intake (SI) is one of the three primary dietary risk factors [1]. A daily SI of about 2 grams can meet the physiological needs of adults. While in fact, SI is currently high in different parts of the world [2, 3], so the World Health Organization recommends population-wide reductions in SI [4]. Numerous studies have demonstrated a causal relationship between excessive SI and essential hypertension and cardiovascular diseases [5–9]. In addition, massive salt restriction experiments and clinical research have found that the reduction of SI not only reduces blood pressure (BP) but also alleviates arterial stiffness, which is independent of the antihypertensive effect, suggesting that salt load may directly affect arterial stiffness [10–14].

RETRACTED

A meta-analysis of 11 randomized controlled trials based on salt restriction in different populations revealed that an average reduction of 89.3 mmol/day in sodium intake was associated with a 2.84% reduction in pulse wave velocity (PWV; 95% CI: 0.51-5.08) [15], but the number of people included was generally small. Based on the Kailuan Study, this research further explored the relationship between perceived SI and arterial stiffness in northern China.

## 2. Participants and Methods

### 2.1. Participants

The data used were from the Kailuan Prospective Cohort Study (Registration No. ChiCTR-TNRC-11001489), an ongoing research project investigating the risk factors and interventions of cardiovascular-related diseases in a functional community population that began in 2006. From 2006 to 2007, a total of 1,015,10 participants (81,110 males and 20,400 females, aged 18–98) received the first health survey composed of questionnaires (e.g., demographic characteristics, chronic diseases, drug use, and lifestyle factors), physical examinations, and laboratory tests at Kailuan General Hospital or its 11 affiliated hospitals. Follow-up was conducted every two years, and brachial-ankle pulse wave velocity (baPWV) testing was started since 2010 (the second follow-up) for some of the observed subjects. All doctors and nurses received rigorous uniform training prior to the study.

In this study, we selected 44,911 people who participated in the follow-up in or after 2010 and completed baPWV detection as observation subjects. Of them, 3991 participants with defective perceived SI data in the questionnaire, 2 with history of atrial flutter and atrial fibrillation, 2943 with chronic kidney disease whose estimated glomerular filtration rate (eGFR) <60 mL/(min·1.73m^2^) or serum creatinine >133 *μ*mol/L, and 1651 with ankle-brachial index (ABI) <0.9 were excluded. Finally, 36,324 subjects were enrolled.

The Ethics Committee at the Kailuan General Hospital approved this study, which strictly followed the principles of the Declaration of Helsinki. Informed consent was obtained from all participants.

### 2.2. SI Assessment

In the questionnaire survey, the participants were asked to assess their perceived SI, so as to rate their daily habitual SI as low, moderate, or high. It has been previously verified in the cohort that the 24-hour urinary sodium excretion corresponding to the perceived SI of the three groups is <6 g (2400 mg/d sodium intake), 6-10 g (2400-4000 mg/d sodium intake), and>10 g (4000 mg/d sodium intake), respectively. For more information, please see the published literature on this topic [16, 17].

RETRACTED

### 2.3. Assessment of Arterial Stiffness

baPWV values were collected by BP-203RPEIII networked arteriosclerosis detection device purchased from OMRON Healthcare (China). Before the test, all participants were prohibited from smoking and asked to rest quietly at room temperature for ≥15 min. During the test, they were asked to lie flat with their pillows removed and keep quiet. The measurement was repeated twice. We collected the larger values of both left and right baPWV and averaged the values of two measurements for analysis. Arterial stiffness was diagnosed if baPWV ≥1400 cm/s [18].

### 2.4. Evaluation of Potential Covariates

#### 2.4.1. Laboratory Indicators

In the morning, about 5 mL of cubital venous blood after 8-12 h of fasting was collected from each participant into a vacuum tube added with ethylenediaminetetra-acetic acid (EDTA). Biochemical indices including serum total cholesterol (TC), low- and high-density cholesterol lipoprotein (LDL-C/HDL-C), and fasting blood glucose (FBG) were detected using a Hitachi 747 automatic analyzer (Tokyo, Japan). eGFR was calculated by referring to the formula of modification of diet in renal disease (MDRD): eGFR=175×[serum creatinine (mg/dl)]^−1.234^ × [age (years)]^−0.179^ × (female × 0.79), unit of calculation mL/(min · 1.73 m^2^) [19].

#### 2.4.2. Physical Examination Indicators

During measurement, the height of the observed subjects was accurate to 0.1 cm and the weight to 0.1 kg. Body mass index (BMI) = weight (kg)/height^2^ (m^2^). Before measurement, the subjects were asked to empty the bladder, not to smoke, and rest quietly for at least 15 min. Before 2014, the right brachial artery BP was determined using a corrected desktop mercury sphygmomanometer (Yuwell, China). The systolic blood pressure (SBP) reading and diastolic blood pressure (DBP) reading took the first and fifth Korotkoff sound, respectively. The measurement was carried out three times continuously with an interval of 1-2 min, and the average value was taken as the measurement result. After 2014, HEM-8102A electronic sphygmomanometer produced by ORMON (Dalian) was used for BP measurement.

#### 2.4.3. Questionnaire Survey Indicators

The trained investigators made face-to-face inquiries and filled in the questionnaire, investigating the participant's basic information such as age, gender, living habits (smoking, drinking, physical labor, and diet), and diseases (hypertension, hyperlipidemia, diabetes, and myocardial infarction). Diagnostic criteria and definitions of related data are detailed in the published literature [20, 21].

RETRACTED

### 2.5. Statistical Methods

SAS statistical software (Version 9.4; SAS Institute, Cary, NC) was responsible for all statistical analyses. Two-tailed *P* < 0.05 suggests the presence of statistical significance.

Normally distributed quantitative data were denoted by mean ± standard deviation ($\bar{X}\pm S$), and skewed distributed ones were represented by median (*P*_25−_*P*_75_). Categorical data was expressed in the form of frequency and percentage (%). One-way ANOVA was used for continuous variables, and *χ*^2^ test was adopted for categorical variables to compare the baseline characteristics of the observed subjects. Besides, we examined the normality of age, SBP, FBG, BMI, TC, and eGFR and found that none of them were normally distributed, so we converted them into classified variables for further analysis. SBP, FBG, TC, and eGFR were converted into categorical variables based on quartiles. Age was classified according to <45, 45-60, 60-75, and>75 years old. And BMI was classified into the following four groups by referring to the Guidelines for the Prevention and Control of Overweight and Obesity in Chinese Adults: <18.5 kg/m^2^: low body weight; 18.5-23.9 kg/m^2^: normal body weight; 24.0-27.9 kg/m^2^: overweight; and ≥28.0 kg/m^2^: obesity.

In order to analyze the association between SI and arterial stiffness, the relationship between SI and baPWV was analyzed using the multiple logistic regression model with perceived SI as the independent variable and arterial stiffness (baPWV ≥1400 cm/s) as the dependent variable. In the analysis of model 1, adjustments were made for gender and age; SBP, BMI, FBG, eGFR, and TC were further adjusted in model 2 based on model 1. And on the basis of model 2, model 3 further adjusted long-term physical labor, smoking, drinking, use of antihypertensive drugs, and use of lipid-lowering agents. Considering that the Dietary Approaches to Stop Hypertension (DASH) diet recommends a daily SI of no more than 6 g [22], people with 6-10 g (moderate SI) and >10 g (high SI) were combined as binary variables and repeated into the multivariate Logistic regression model.

## 3. Results

### 3.1. Clinical Data

Among the 36,324 subjects, 25,934 were males (71.40%) and 10,390 were females (28.60%), with a mean age of 49.10 ± 12.57 years, an average baPWV of 1527.73 ± 355.61 cm/s, and a baPWV ≥1400 cm/s percentage of 57.57%. All subjects were divided into three (low, medium, and high) SI groups according to their perceived SI.

The baseline characteristics of the observed objects classified according to perceived SI are shown in Table 1. The number of people in the medium SI group was the largest, accounting for 77.51%, followed by the low SI group, with the number of cases in the high SI group being the lowest. The three groups were nonsignificantly different in sex, age, SBP, DBP, BMI, FBG, TC, HDL-C, eGFR, smoking, drinking, and prevalence of hypertension, hyperlipidemia, diabetes mellitus, and myocardial infarction (*P* < 0.05). The male ratio, SBP, DBP, FBG, TC, and average baPWV were significantly higher in the high SI group compared with medium and low SI groups, as well as the prevalence of arterial stiffness (baPWV ≥1400 cm/s), hypertension, hyperlipidemia, diabetes, and myocardial infarction.

RETRACTED

### 3.2. Logistic Regression Analysis

Variable assignments for logistic regression analysis are shown in Table 2. The adjusted odds ratios (ORs) and 95% confidence intervals (CIs) for different perceived SI groups can be found in Table 3. After adjusting for sex, age, related laboratory indexes, lifestyle factors, and medication, moderate SI and high SI were found to be statistically correlated with baPWV ≥1400 cm/s (*P* < 0.05), with the OR and 95% CI of 1.11 (1.03-1.19) and 1.17 (1.04-1.31), respectively.

With the low SI population as the reference, the medium and high SI population were combined and repeated into the multivariate logistic regression model, as shown in Table 4. It showed that perceived SI ≥6 g was statistically associated with arterial stiffness (baPWV ≥1400 cm/s) (*P* < 0.05), with an OR (95% CI) of 1.11 (1.03-1.20).

## 4. Discussion

In previous studies, age, sex, FBG, and SBP were identified as independent risk factors for arterial stiffness, which were also verified in our research [23–27]. In the presented study, we explored the association of perceived SI with arterial stiffness in northern China and found that perceived SI ≥ 6 g was also the risk factor for arterial stiffness.

Arterial stiffness is a pathological process of the structure and function of the arterial wall that changes mainly with age, as well as the pathological basis of cardio-cerebrovascular events [28], but its specific pathogenesis is not completely clear. In addition to age, most current views believe that persistent elevated BP is the direct cause of increased arterial stiffness, so studies linking salt or sodium to arterial stiffness have been limited to untreated hypertension. Han [29] et al. studied the relationship between urine sodium, urinary sodium-to-potassium (Na/K) ratio, and arterial stiffness in 224 hypertensive patients who did not take antihypertensive drugs. The results showed that urinary sodium and urinary Na/K ratio were independently related to baPWV. However, similar results could not explain the occurrence of arterial stiffness in patients with normal BP. This study included a general population with hypertension, diabetes, hyperlipidemia, or myocardial infarction, and similar results were obtained after adjustment for relevant confounders and medication history.

RETRACTED

Affected by dietary habits, the per capita SI in China is higher than the global average, especially in northern China [30]. In our study, the risk of arterial stiffness increased as SI increased. Compared with low SI, the risk of arterial stiffness is 1.11 times higher with medium SI and 1.17 times higher with high SI. The results indicated that high SI might result in increased risk of arterial stiffness. Therefore, limiting SI is particularly important for the prevention and treatment of arterial stiffness among people with preference for salty tastes.

In addition, Luis et al. found a J-shaped curve when investigating the association between arterial stiffness and sodium intake quartile level, similar to the J-shaped curve between SI and CVD [6–8, 31]. In this study, although the prevalence of hypertension, myocardial infarction, hyperlipidemia, and diabetes was lower in the moderate SI population than that in the low SI population, the measurement value of baPWV and the proportion of arterial stiffness (baPWV ≥1400 cm/s) did not increase significantly, which indicated that extremely low SI may mean a higher risk of arterial stiffness. However, it may also be related to the relatively high SI in the study population.

Dietary habits of different races and regions, as well as a not-yet-agreed method of calculating sodium salt, could all contribute to inconsistent results. Strauss et al. studied 693 adults aged 20 to 30 years, 51% of whom were black, and found that the association between SI and baPWV was significant in young, healthy blacks, but not in whites [12]. The average SI in northern China is higher than that in other parts of the world [30], so the influence of SI on BP and arterial stiffness in this study is more significant. Currently, the most accurate way to define SI in epidemiological studies is to extrapolate it from 24-hour urine samples [32]. However, this method is time-consuming and costly and is therefore not suitable for large-scale samples [33]. In this paper, a small sample was used to verify that there were significant differences in 24-hour urinary sodium excretion among people with different taste preferences. Therefore, the assessment of taste preferences can basically reflect the level of SI. baPWV, while not the golden standard for arterial stiffness, correlates well with the Framingham risk score [24] and is considered a good predictor of cardiovascular events and all-cause mortality [18, 34, 35].

RETRACTED

There are also some shortcomings in this paper. The research population of this study is limited to the in-service and retired employees of the Kailuan Group with their routine physical examination data as the baseline data, which has certain geographical limitations and population selection bias. Second, taste perception is affected by various factors, and the use of perceived SI to determine SI level is not as accurate as 24-hour urine sodium or urine Na/K ratio, especially for the elderly with hypogeusia, as well as those who smoke, drink tea, and/or take medicine for a long time. Finally, this study was cross-sectional and could not assess the long-term effects of changes in SI on arterial stiffness. In the future, a prospective study can be designed based on the above results to further explore whether changes in salty taste have an effect on arterial stiffness.

## Figures and Tables

**Table 1:** Comparison of general data of people with salt preference ($\bar{X}\pm S$, *n* = 36324).

	< 6 g	6-10 g	> 10 g	*F*/*χ*^2^	*P*
	(*n* = 5230)	(*n* = 28153)	(*n* = 2941)		
Male [*n*(%)]	3722 (71.17)	19865 (70.56)	2347 (79.80)^ab^	111.53	<0.01
Age (years)	49.65 ± 12.63	48.87 ± 12.86^a^	50.30 ± 12.22^ab^	22.27	<0.01
SBP (mmHg)	133.40 ± 20.28	132.75 ± 20.05	134.94 ± 20.89^ab^	16.78	<0.01
DBP (mmHg)	82.47 ± 11.38	81.90 ± 11.37^a^	84.42 ± 11.71^ab^	67.07	<0.01
BMI (kg/m^2^)	24.97 ± 3.36	25.10 ± 3.43	25.62 ± 3.52^ab^	36.62	<0.01
FBG (mmol/L)	5.82 ± 1.75	5.77 ± 1.73^a^	5.88 ± 1.79^b^	6.37	<0.01
HDL-C (mmol/L)	1.50 ± 0.54	1.47 ± 0.45^a^	1.47 ± 0.43	10.42	<0.01
LDL-C (mmol/L)	2.82 ± 0.83	2.78 ± 0.85^a^	2.82 ± 0.88^b^	6.04	0.02
TC (mmol/L)	4.81 ± 1.30	4.89 ± 1.16	4.94 ± 1.25^ab^	14.53	<0.01
eGFR [ml/(min · 1.73 m)]	110.84 ± 47.20	115.20 ± 59.25^a^	111.32 ± 53.03^b^	16.99	<0.01
baPWV (cm/s)	1519.17 ± 346.25	1518.40 ± 351.05	1559.16 ± 361.07^ab^	18.11	<0.01
baPWV ≥1400 cm/s [*n* (%)]	2954 (56.48)	15882 (56.41)	1827 (62.12)^ab^	35.79	<0.01
Long-term manual labor [*n* (%)]	4647 (88.85)	25127 (89.25)	2626 (89.29)	0.76	0.68
Smoking [*n* (%)]	2416 (46.20)	13113 (46.58)	1699 (57.77)^ab^	137.5	<0.01
Drinking [*n* (%)]	994 (19.01)	5063 (17.98)	767 (26.08)^ab^	114.58	<0.01
History of hypertension [*n* (%)]	2037 (38.95)	10227 (36.33)^a^	1268 (43.11)^ab^	60	<0.01
History of hyperlipidemia [*n* (%)]	388 (7.42)	1516 (5.38)^a^	288 (9.79)^ab^	111.88	<0.01
History of diabetes [*n* (%)]	603 (11.53)	3095 (10.99)	413 (14.04)^ab^	24.94	<0.01
History of myocardial infarction [*n* (%)]	70 (1.34)	282 (1.00)	37 (1.26)	5.78	<0.01
Use of antihypertensives [*n* (%)]	927 (17.72)	4432 (15.74)^a^	646 (21.97)^ab^	81.03	<0.01
Use of lipid-lowering agents [*n* (%)]	59 (1.13)	170 (0.60)^a^	33 (1.12)^b^	24.11	<0.01

Note: Normally distributed measurement data is expressed as ($\bar{X}\pm S$), and the skewed distributed ones are represented by median (*P*_25_ − *P*_75_). SBP: systolic blood pressure; DBP: diastolic blood pressure; BMI: body mass index; FBG: fasting blood glucose; baPWV: brachial-ankle pulse wave velocity; TC: total cholesterol; HDL-C: high-density lipoprotein cholesterol; LDL-C: low-density lipoprotein cholesterol. 1 mmHg = 0.133 kPa. ^a^Indicates *P* < 0.05 compared with the <6 g group; ^b^Indicates *P* < 0.05 compared with the 6-10 g group.

RETRACTED

**Table 2:** Variable assignment of multivariate logistic regression analysis.

Variable	Assignment
Salt intake	0: low salt intake; 1: medium salt intake; 2: high salt intake
Sex	0: female; 1: male
Age	0: age < 45; 1: 45 ≤ age <60; 2: 60 ≤ age < 75; 3: age ≥ 75
Systolic blood pressure (SBP)	0: SBP < *P*_25_; 1: *P*_25_≤ SBP < *P*_50_; 2: *P*_50_≤ SBP < *P*_75_; 3: SBP ≥ *P*_75_
Body mass index (BMI)	0: BMI <18.5; 1: 18.5 ≤ BMI < 24; 2: 24 ≤ BMI < 28
Fasting blood glucose (FBG)	0: FBG <*P*_25_; 1: *P*_25_≤ FBG < *P*_50_; 2: *P*_50_< FBG < *P*_75_; 3: FBG ≥*P*_75_
eGFR	0: eGFR < *P*_25_; 1: *P*_25_≤ eGFR < *P*_50_; 2: ≤ eGFR < *P*_75_; 3: eGFR > *P*_75_
Total cholesterol (TC)	0: TC < *P*_25_; 1: *P*_25_≤ TC < *P*_50_; 2: *P*_50_≤ TC < *P*_75_; 3: TC ≥ *P*_75_
Long-term manual labor	0: no; 1: yes
Smoking	0: no; 1: yes
Drinking alcohol	0: no; 1: yes
Use of antihypertensives	0: no; 1: yes
Use lipid-lowering agents	0: no; 1: yes

**Table 3:** Factors influencing brachial-ankle pulse wave velocity by multivariate Logistic regression analysis (*n* = 36324).

Variable	Model 1		Model 2		Model 3	
	OR (95% CI)	*P*	OR (95% CI)	*P*	OR (95% CI)	*P*
<6 g	1.00		1.00		1.00	
6-10 g	1.05 (0.98-1.13)	0.14	1.10 (1.02-1.18)	0.01	1.11 (1.03-1.19)	<0.01
>10 g	1.16 (1.04-1.29)	<0.01	1.20 (1.07-1.35)	<0.01	1.17 (1.04-1.31)	<0.01
Sex	3.14 (2.98-3.32)	<0.01	2.03 (1.91-2.16)	<0.01	1.96 (1.82-2.11)	<0.01
Age	4.21 (4.06-4.36)	<0.01	3.20 (3.08-3.33)	<0.01	3.05 (2.93-3.17)	<0.01
Systolic blood pressure	—	—	2.09 (2.04-2.14)	<0.01	1.95 (1.90-2.00)	<0.01
Body mass index	—	—	0.94 (0.90-0.97)	<0.01	0.92 (0.89-0.96)	<0.01
Fasting blood glucose	—	—	1.21 (1.18-1.24)	<0.01	1.21 (1.18-1.24)	<0.01
eGFR	—	—	0.98 (0.96-1.00)	0.10	0.98 (0.96-1.00)	0.09
Total cholesterol	—	—	1.12 (1.09-1.14)	<0.01	1.12 (1.09-1.14)	<0.01
Long-term manual labor	—	—	—	—	1.44 (1.31-1.57)	<0.01
Smoking	—	—	—	—	1.05 (0.99-1.12)	0.13
Drinking	—	—	—	—	1.10 (1.02-1.19)	<0.01
Use of antihypertensives	—	—	—	—	1.95 (1.77-2.15)	<0.01
Use of lipid-lowering agents	—	—	—	—	0.99 (0.70-1.42)	0.97

Note: model 1: adjusted for age and sex; model 2: systolic blood pressure, body mass index, fasting blood glucose, estimated glomerular filtration rate, and total cholesterol were adjusted on the basis of model 1; model 3: regular exercise, smoking, drinking, used of antihypertensives, and lipid-lowering agents were adjusted on the basis of model 2.

RETRACTED

**Table 4:** Factors influencing brachial-ankle pulse wave velocity by multivariate Logistic regression analysis (sensitivity analysis, *n* = 36324)∗.

Variable	Model 1		Model 2		Model 3	
	OR (95% CI)	*P*	OR (95% CI)	*P*	OR (95% CI)	*P*
<6 g	1.00		1.00		1.00	
>6 g	1.09 (1.03-1.17)	0.01	1.13 (1.05-1.22)	<0.01	1.11 (1.03-1.20)	<0.01
Sex	3.15 (2.98-3.33)	<0.01	2.08 (1.96-2.21)	<0.01	1.96 (1.83-2.11)	<0.01
Age	1.11 (1.107-1.113)	<0.01	1.09 (1.088-1.093)	<0.01	3.05 (2.93-3.17)	<0.01
Systolic blood pressure	—	—	2.05 (1.99-2.10)	<0.01	1.95 (1.89-2.00)	<0.01
Body mass index	—	—	0.95 (0.92-0.99)	0.01	0.92 (0.89-0.96)	<0.01
Fasting blood glucose	—	—	1.18 (1.15-1.21)	<0.01	1.21 (1.18-1.24)	<0.01
eGFR	—	—	1.02 (0.99-1.04)	0.18	0.98 (0.96-1.00)	0.09
Total cholesterol	—	—	1.09 (1.06-1.11)	<0.01	1.12 (1.09-1.14)	<0.01
Long-term manual labor	—	—	—	—	1.44(1.31-1.57)	<0.01
Smoking	—	—	—	—	1.05 (0.99-1.12)	0.12
Drinking	—	—	—	—	1.10 (1.03-1.19)	<0.01
Use of antihypertensives	—	—	—	—	1.96 (1.77-2.16)	<0.01
Use of lipid-lowering agents	—	—	—	—	1.00 (0.70-1.42)	0.98

Note: ∗Combining moderate salt intake with high salt intake population. Model 1: adjusted for age and sex; model 2: systolic blood pressure, body mass index, fasting blood glucose, estimated glomerular filtration rate, and total cholesterol were adjusted on the basis of model 1; model 3: based on model 2, regular exercise, smoking, drinking, use of antihypertensives, and use of lipid-lowering agents were further adjusted.

## Data Availability

The labeled dataset used to support the findings of this study are available from the corresponding author upon request.
